# The Clinical Application of Remimazolam Benzenesulfonate Combined with Esketamine Intravenous Anesthesia in Endoscopic Retrograde Cholangiopancreatography

This article has been retracted.

**DOI:** 10.1155/2022/5628687

**Published:** 2022-06-30

**Authors:** Xiuna Yi, Weiwei Xu, Aizhi Li

**Affiliations:** ^1^Department of Anesthesiology, Yantaishan Hospital, Yantai, 264003 Shandong, China; ^2^Department of Anesthesiology, Yuhuangding Hospital, Yantai, Shandong 264000, China

## Abstract

In this project, algorithm-based image processing methods in 3D endoscopic image processing endoscopic retrograde cholangiopancreatography (ERCP) were analyzed. To enhance local information of images, an adaptive histogram equalization method with limited contrast is introduced. The influences of the algorithm on 3D endoscopic image peak signal-to-noise ratio (PSNR), image discrete information entropy (DE), and average mean brightness error (AMBE) of images before and after the optimization before were compared. A total of 92 patients receiving ERCP at Yuhuangding Hospital between December 2019 and December 2021 were selected and divided into the control group (fentanyl+propofol) and the observation group (remimazolam benzenesulfonate+esketamine). Mean arterial pressure heart rate (HR), oxygen saturation (SpO_2_), and respiratory rate (RR) of the patients at each time point including the entry into the operation room (T0), 2 minutes after the beginning of medication (T1), after endoscopy (T2), endoscopy withdrawal (T3), and postoperative awakening (T4) were recorded. The comparison of MAP between T1, T2, T3, and T4 and T0 among patients in the observation group and the control group showed statistical differences (*P* < 0.05). Besides, HR and RR at T4 in the observation group were obviously higher than those in the control group (*P* < 0.05). The comparison of SpO_2_ at T3 and T4 and that at T0 both showed statistical differences (*P* < 0.05). Awakening time and VAS scores in the observation group were obviously lower than those in the control group (*P* < 0.05). The incidence of bradycardia, nausea, vomiting, and chill in the observation group was all lower than that in the control group (*P* < 0.05). The results indicated that an effective endoscopic image processing method was established based on an image enhancement algorithm, and the combination of remimazolam benzenesulfonate and esketamine showed high safety and efficacy in ERCP.

## 1. Introduction

Endoscopic retrograde cholangiopancreatography (ERCP) is one of the commonly used means of the examination and treatment of pancreatic bile tract and gall bladder. ERCP is featured with minor trauma, accurate efficacy, and short postoperative hospitalization stay [1] and is widely applied in the clinical diagnosis and treatment of pancreas and bile duct systems. However, more and more clinical studies reveal that nausea, vomiting, cardiovascular stress reaction, and unstable hemodynamics are caused during the operation of ERCP. Severe patients suffer from respiratory and circulatory dysfunctions, resulting in emergency conditions [2–4]. Clinically, sedative drugs and analgesic drugs are often adopted in combination to ensure spontaneous breathing of patients, maintain stable hemodynamics, and avoid respiratory suppression [5]. At present, the anesthesia scheme used clinically can generally meet the diagnosis and treatment of ERCP, but adverse reactions still occur [6]. Esketamine is a new anesthetic sedative and analgesic drug, which is featured with quick effects, short duration, and high controllability. It does not inhibit respiratory and circulation systems. However, the use of esketamine alone causes nausea, vomiting, and seizures [7]. Remimazolam benzenesulfonate is a benzodiazepine sedative hypnotic, which can reduce the excitability of neurons and is characterized by a fast effect, short awakening time, and minor influence on the body circulation system [8]. Nevertheless, it shows no sedative effect and can only be used together with other narcotic analgesics. Some researchers applied remimazolam benzenesulfonate combined with propofol in painless induced abortion. The results demonstrated a low incidence of injection pain, mild inhibition of respiratory circulation, and higher quality of awakening [9]. At present, there are few studies on the combination of esketamine and remimazolam benzenesulfonate in anesthesia. Besides, its efficacy and security are both unknown.

Endoscopy is an instrument commonly used in the clinical diagnosis and treatment of different diseases. 3D endoscopy can obtain left and right binocular views to offer 3D information about objects and significantly improve the accuracy of disease diagnosis and treatment. The 3D endoscopy image acquisition environment is dim and dark. The artificial addition of light source and color temperature has obvious influences on image colors. Besides, thermal noise exists in the image acquisition device, which causes a series of noises in endoscopic images, such as pulse noise and salt and pepper noise. In the processes of acquiring and transmitting endoscopic images, color deviation and image quality degeneration also come into being [10, 11]. Hence, 3D endoscopic image processing should not only consider the color and quality of images but also need to focus on the consistency of the colors of left and right binocular images. Traditional endoscopic processing algorithms include the image enhancement algorithm and the image white balance algorithm [12]. They can effectively enhance endoscopic images. The wavelength transformation-based image enhancement algorithm can enhance the local contrast ratio and shows significant effects on image defogging and denoising. Nonetheless, there are still some disadvantages in actual application, such as excessive amplification of noises and large computation [13]. It needs to be further optimized.

To sum up, there are few studies on the combination of esketamine and remimazolam benzenesulfonate in anesthesia, and its efficacy and security are both unknown. The image enhancement algorithm in 3D endoscopic image processing still needs to be further optimized. Hence, endoscopic images are processed, and the efficacy and security of remimazolam benzenesulfonate combined with esketamine intravenous anesthesia in ERCP were discussed based on the image enhancement algorithm. The discussion provided a reference direction and some guiding significance for 3D endoscopic image processing and ERCP anesthesia scheme.

## 2. Materials and Methods

### 2.1. Image Enhancement Algorithm-Based 3D Endoscopic Image Method

In terms of the wavelet transformation-based image enhancement algorithm, there are some disadvantages in image enhancement processing, including low local contrast ratio and incomplete processing of high-frequency images. Based on the wavelet transformation image enhancement algorithm, the local image information about low-frequency parts was enhanced by an adaptive histogram equalization method with limited contrast. Besides, the homomorphic filtering enhancement algorithm was introduced for filter processing. The Sobel gradient operator was adopted to sharpen the edges of high-frequency parts in images.  Figure 1 displays the image processing procedures by the wavelet transformation-based image enhancement algorithm.

Two-dimensional wavelet transformation can reduce the dimension of images by horizontal and vertical filtering. The Mallat algorithm is a fast wavelet decomposition method by which endoscopic images are filtered horizontally and vertically. After the dimensionality reduction, the images are decomposed into four subgraphs, including low-frequency components, horizontal high frequency, vertical high frequency, and diagonal high-frequency components [14]. After wavelet reconstruction, each subgraph is synthesized. The Mallat algorithm image decomposition algorithm is expressed by

(1) $$\begin{array}{c} A_{i+1}\left(n\right)=\underset{k}{\sum }G\left(k\right)A_{i}\left(2n-k\right), \end{array}$$

(2) $$\begin{array}{c} B_{i+1}\left(n\right)=\underset{k}{\sum }F\left(k\right)A_{i}\left(2n-k\right). \end{array}$$

In equations (1) and (2), *G*(*k*) and *F* (*k*) denote low-pass filters and high-pass filters, respectively.

Homomorphic filtering enhancement is a standard image enhancement technology mainly applied in the processing of the image frequency domain [15]. Hence, the Fourier transform is adopted to convert endoscopic images into the frequency domain. In addition, a high-pass homomorphic filter is introduced to inhibit low-frequency parts and enhance high-frequency parts. The algorithm of the homomorphic filter for image enhancement is expressed by

(3) $$\begin{array}{c} E\left(\alpha ,\varepsilon \right)=H_{i}\left(\alpha ,\varepsilon \right)I\left(\alpha ,\varepsilon \right)+H_{j}\left(\alpha ,\varepsilon \right)I\left(\alpha ,\varepsilon \right). \end{array}$$

In equation (3), *H* (*α*, *ε*) refers to the high-pass homomorphic filter and *I* (*α*, *ε*) indicates the pixel value at the coordinate of (*α*, *ε*).

After homomorphic filtering enhancement, the inverse discrete Fourier transform is adopted. The image is transformed into a spatial image, and its calculation method is expressed by

(4) $$\begin{array}{c} e\left(x,y\right)=H^{-1}\left[H_{i}\left(\alpha ,\varepsilon \right)I\left(\alpha ,\varepsilon \right)+H_{j}\left(\alpha ,\varepsilon \right)I\left(\alpha ,\varepsilon \right)\right]. \end{array}$$

The quality of endoscopic images is correlated with the degree of the light source. An appropriate high-pass homomorphic filter is required for reducing the weakening of image quality caused by uneven illumination [16]. The Gaussian high-pass filter is one of the commonly used homomorphic filters. Its calculation method is expressed by

(5) $$\begin{array}{c} I\left(\alpha ,\varepsilon \right)=\left(jI-jL\right)\left[1-\frac{-{mD}^{2}\left(\alpha ,\varepsilon \right)}{e^{D_{0}^{2}}}\right], \end{array}$$

(6) $$\begin{array}{c} D\left(\alpha ,\varepsilon \right)={\left[{\left(\alpha -\frac{m}{2}\right)}^{2}-{\left(\varepsilon -\frac{n}{2}\right)}^{2}\right]}^{1/2}. \end{array}$$

In equations (5) and (6), *jI* refers to high-frequency gain, *jL* denotes low-frequency gain, *D*(*α*, *ε*) represents the distance from the frequency (*α*, *ε*) to the filter center, and *D*_0_ indicates cutoff frequency. A large number of studies verify that *jI* is finally set as 7 and *jL* is set to be 0.5 in the research.

The adaptive histogram equalization method with limited contrast is a histogram equalization processing after the segmentation of images into blocks. It shows a very significant processing effect on the images with extensive pixel distribution [17]. Besides, the bilinear interpolation method was adopted to avoid the incidence of the block effect [18].  Figure 2 shows the specific processes of the adaptive histogram equalization with limited contrast.

Median filtering is an effective nonlinear filtering technique for image protection [19]. During the window sliding process, window width cannot be obtained at the edge. 0 is adopted to fill the window width. After that, the window width is sorted, and the median is taken. The calculation method of median filtering is expressed by

(7) $$\begin{array}{c} Z_{i,j}=\text{Med}\left(X_{i,j}\right). \end{array}$$

High-frequency images need to be sharpened. The Sobel operator obtains the approximate value of image brightness function grayscale by the gradient scale method for the sharpening [20]. The convolution factor of the Sobel gradient operator is expressed by

(8) $$\begin{array}{c} J_{x}=\left[\begin{array}{ccc} -1 & 0 & 1\\ -2 & 0 & 2\\ -1 & 0 & 1 \end{array}\right]*I, \end{array}$$

(9) $$\begin{array}{c} J_{y}=\left[\begin{array}{ccc} 1 & 2 & 1\\ 0 & 0 & 0\\ -1 & -2 & -1 \end{array}\right]*I. \end{array}$$

In equations (8) and (9), *J*_*x*_ and *J*_*y*_ represent the pixel values of the images after the horizontal and vertical edge detection, respectively.

The image pixel value after the sharpening of the Sobel gradient operator is expressed by

(10) $$\begin{array}{c} J=\sqrt{J_{x}^{2}+J_{y}^{2}}. \end{array}$$

### 2.2. Evaluation Indexes of Endoscopic Images

The processed endoscopic images are evaluated by the peak signal-to-noise ratio (PSNR), image discrete information entropy (DE), and average mean brightness error (AMBE). The calculation method of PSNR is expressed by

(11) $$\begin{array}{c} \text{PSNR}=10\log\left(\frac{{\left(L-1\right)}^{2}}{\text{MSE}}\right), \end{array}$$

(12) $$\begin{array}{c} \text{MSE}=\frac{1}{N}\underset{i=1}{\sum }\underset{j=1}{\sum }{\left\|X\left(i,j\right)-Y\left(i,j\right)\right\|}^{2}. \end{array}$$

In equations (11) and (12), *L* refers to the maximum value of image pixel, *N* denotes the number of image pixel points, *X*(*i*, *j*) represents the grayscale of input images, and *Y*(*i*, *j*) indicates the grayscale of output images.

DE is often used for the assessment of the richness of image details. A greater DE means richer image details. Its calculation method is shown in

(13) $$\begin{array}{c} \text{DE}=\overset{L-1}{\underset{i=0}{\sum }}P_{y}\left(i\right)\log2P_{y}\left(i\right). \end{array}$$

In equation (13), *P*_*y*_(*i*) refers to the probability density of gray level *i*.

AMBE assesses the errors in the absolute brightness of images before and after the processing. A smaller AMBE indicates a better image enhancement effect:

(14) $$\begin{array}{c} \text{AMBE}=\left|M\left(X\right)-M\left(Y\right)\right|. \end{array}$$

In equation (14), *M*(*X*) and *M*(*Y*) represent the average brightness of input and output images, respectively.

### 2.3. Research Objects and Grouping

A total of 92 patients receiving ERCP at Yuhuangding Hospital between December 2019 and December 2021 were selected as the research objects, including 63 males and 29 females. The patients were aged between 60 and 86 with an average of 67.84 ± 5.97. The patients were included based on the following criteria.

- Patients who were above 60 years old
- Patients with the American Society of Anesthesiologists (ASA) grade [21] between levels I and III
- Patients without a history of drug allergy
- Patients without abnormal renal function and history of hypertension
- Patients without arrhythmia

The patients were excluded based on the following criteria.

- Patient with a history of malignant high fever family
- Patients allergic to drugs
- Patients who took benzodiazepine drugs or opiates in the last 3 months
- Patients with respiratory diseases or difficult airways
- Patients with a family history of mental diseases
- Patients with bradycardia or atrioventricular block
- Patients with anemia history

All included research objects were divided into the control group (fentanyl+propofol) and the observation group (remimazolam benzenesulfonate+esketamine) by the random number table method. There were 46 cases in each group. The patients in the two groups were performed with intravenous anesthesia. The process of the experiment had been approved by the Yuhuangding Hospital Ethics Committee, and all included research objects had signed the informed consent forms.

### 2.4. ERCP Anesthesia Methods

All patients were ordered to fast for 24 hours and refrained from drinking for 8 hours before the operation. On the day of the operation, patients needed to take 0.25 mg alprazolam orally after getting up. All endoscopic operations were performed by 3 senior attending physicians in the department of gastroenterology of the hospital, and 1 senior anesthesia attending physician carried out the anesthesia. After the patients entered the operation room, 500 mL acetic acid Ringer's injection was intravenously dropped from the outer limb. Patients were asked to lie on their sides and uptake oxygen at 4 L/min with a nasal catheter. The patients in the control group were injected with 1 mg/kg propofol (Xi'an Libang Management Co., Ltd., H20010368) and 1 *μ*g/kg fentanyl (Yichang Humanwell Pharmaceutical Co., Ltd., H20054171) intravenously. 0.4 mg/kg remimazolam benzenesulfonate (Yichang Humanwell Pharmaceutical Co., Ltd.) and 1 mg/kg esketamine (Jiangsu Hengrui Pharmaceuticals Co., Ltd.) were injected intravenously into the patients in the observation group. When the Ramsay score reached 5 points, endoscopy was performed. The patients in the control group were performed intravenous pump injection of 12 *μ*g/(kg·h) fentanyl and 4 mg/(kg·h) propofol as the maintenance medication. The patients in the observation group received the intravenous pump injection of 1 mg/(kg·h) remimazolam benzenesulfonate and 0.5 mg/(kg·h) esketamine. Based on the bispectral index (BIS), the dosage of narcotics was adjusted. When the endoscope was withdrawn, anesthesia pumping was stopped to improve the Aldrete score as sober scoring criteria. After the patients awoke, they were observed for 30 minutes and then escorted back to the ward.

### 2.5. Observation Indexes

The visual analogue scale (VAS) [22] was adopted to assess the degree of pain after the patients awoke. No pain was scored 0 points, mild pain was scored between 1 and 3 points, moderate pain was scored between 4 and 6 points, severe pain was scored between 7 and 9 points, and sharp and unbearable pain was scored 10 points. MAP, HR, SpO_2_, and RR at each time point including the entry into the operation room (T0), 2 minutes after the medication (T1), after endoscopy (T2), endoscopy withdrawal (T3), and postoperative awakening (T4) of patients were recorded. In addition, the statistics on intraoperative respiratory circulation inhibition time of hypotension, bradycardia, decreased SpO_2_, and respiratory suppression among the patients in the two groups was carried out. The incidence of nausea, vomiting, and other postoperative complications of the patients in the two groups were recorded. The differences in VAS scores, operation time, and awakening time after they awoke were compared.

### 2.6. Statistical Methods

Experimental data were processed by statistical product and service solutions (SPSS) 19.0. Measurement data were expressed by the mean ± standard deviation ($\bar{x}\pm \text{s}$) and performed with a *t*-test. Enumeration data were denoted by percentage (%) and performed with the *χ*^2^ test. Besides, *P* < 0.05 indicated that the differences showed statistical significance.

## 3. Results

### 3.1. Analysis of Results of Image Enhancement Algorithm-Based 3D Endoscopic Image Processing

45 endoscopic images were selected randomly and processed with the enhancement algorithm before and after optimization. PSNR values of 3D endoscopic images processed by the enhancement algorithm before and after optimization were compared (Figure 3). The results showed that the PSNR value of the images processed by the optimized enhancement algorithm was obviously higher than that of the enhancement algorithm before optimization.

The enhancement algorithms before and after optimization were adopted to process 3D endoscopic images. DE values of 3D endoscopic images processed by the enhancement algorithms before and after optimization were compared (Figure 4). The results illustrated that the DE value of the images processed by the optimized enhancement algorithm was obviously higher than that processed by the enhancement algorithm before optimization.

The enhancement algorithms before and after optimization were adopted to process 3D endoscopic images. AMBE values of 3D endoscopic images processed by the enhancement algorithms before and after optimization were compared (Figure 5). The results demonstrated that the AMBE value of the images processed by the optimized enhancement algorithm was obviously lower than that processed by the enhancement algorithm before optimization. The AMBE value of the images processed by the optimized enhancement algorithm was obviously lower than those processed by the enhancement algorithm before optimization.

### 3.2. Basic Information about Included Objects

The age, gender proportion, weight, ASA grades, and the proportion of patients diagnosed with different diseases clinically in the two groups were summarized and analyzed (Table 1). The comparison of the above information all showed no statistical differences (*P* > 0.05).

### 3.3. Comparison of Hemodynamics and Respiratory Frequency of the Patients in Two Groups at Different Time Points

MAP of the patients in the observation group and the control group at different time points was compared (Figure 6). The comparison of MAP of the patients in the two groups at T0 showed no statistical differences (*P* > 0.05). From T1, MAP of the patients in the two groups both demonstrated an obvious descending trend. The comparison of MAP of the patients in the observation group and the control group between T1, T2, T3, and T4 and T0 all had statistical differences (*P* < 0.05). Besides, MAP in the observation group at T1, T2, T3, and T4 was obviously higher than those in the control group (*P* < 0.05).

HR of the patients in the observation group and the control group at different time points were compared (Figure 7). The comparison of HR of the two groups at T0 showed no statistical differences (*P* > 0.05). From T1, HR of the patients in the two groups both showed an obvious descending trend. The comparison of HR between at T4 and at T0 in the observation group both had statistical differences (*P* < 0.05). The comparison of HR at T3 as well as T4 and at T0 both showed statistical differences (*P* < 0.05). Besides, HR of the patients in the observation group at T4 was obviously higher than that in the control group at T4 (*P* < 0.05).

RR of the patients in the observation group and the control group at different time points were compared (Figure 8). The comparison of RR of the patients in two groups at T0 showed no statistical differences (*P* > 0.05). From T1, RR of the patients in the two groups both showed an obvious descending trend. The comparison of RR in the observation group at T4 and at T0 both had statistical differences (*P* < 0.05). The comparison of RR at T3 as well as T4 and at T0 both had statistical differences (*P* < 0.05). In addition, RR of the patients in the observation group at T4 was obviously higher than that in the control group at T4 (*P* < 0.05).

SpO_2_ of the patients in the observation group and the control group at different time points were compared (Figure 9). The comparison of SpO_2_ of the patients in the two groups at T0 showed no statistical differences (*P* > 0.05). From T1, SpO_2_ of the patients in the two groups both showed an obvious descending trend. The comparison of SpO_2_ of the patients in the control group at T3 as well as T4 and at T0 both had statistical differences (*P* < 0.05). Besides, SpO_2_ in the observation group at T3 and T4 were obviously higher than those in the control group (*P* < 0.05).

### 3.4. Comparison of Operation Time, Awakening Time, and Postoperative VAS Scores of the Patients in Two Groups

Operation time, awakening time, and VAS scores after the awakening of the patients in the observation group and the control group were compared (Figure 10). The comparison of operation time between the patients in the two groups showed no statistical differences (*P* > 0.05). The awakening time of the patients in the control group and the observation group was 22.51 ± 2.02 minutes and 9.03 ± 1.08 minutes, respectively. Obviously, the awakening time in the observation group was shorter than that in the control group (*P* < 0.05). VAS scores after the awakening of the patients in the control group and the observation group were 3.65 ± 0.33 minutes and 1.98 ± 0.18 minutes, respectively. It was obvious that the VAS score after the awakening in the observation group was lower than that in the control group (*P* < 0.05).

### 3.5. Comparison of the Incidence of Adverse Events and Complications of the Patients in the Two Groups

The incidence of intraoperative adverse events of the patients in the observation group and the control group was compared (Figure 11). The incidence of hypotension, bradycardia, low oxygen saturation, and respiratory suppression in the control group was 8 (17.39%), 6 (13.04%), 13 (28.26%), and 10 (21.74%), respectively. Those in the observation group were 2 (4.35%), 1 (2.17%), 4 (8.70%), and 1 (2.17%), respectively. The results showed that the incidence of hypotension, low oxygen saturation, and respiratory suppression in the observation group were all obviously lower than those in the control group (*P* < 0.01). The comparison of the incidence of bradycardia between the observation group and the control group had statistical differences (*P* < 0.05).

The incidence of postoperative complications of the patients in the observation group and the control group was compared (Figure 12). The incidence of nausea, vomiting, and chill in the control group was 6 (13.04%), 4 (8.70%), and 3 (6.52%), respectively. Those in the observation group were 3 (6.52%), 1 (2.17%), and 1 (2.17%), respectively. The results revealed that the incidence of nausea, vomiting, and chill in the observation group was all lower than those in the control group (*P* < 0.05).

## 4. Discussion

After the processing of the specific information about images through specific algorithms, image enhancement can meet the need of human vision or machine vision [23]. In the research, an adaptive histogram with limited contrast, homomorphic filtering enhancement algorithm, and Sobel gradient operator were introduced to optimize the images based on the image enhancement algorithm. The results showed that PSNR, DE, and AMBE of the optimized algorithm were all obviously superior to those of the algorithm before optimization, which was caused by the targeted improvement of the contrast ratio of the specific areas of images by the introduced adaptive histogram with limited contrast compared with the histogram equalization method [24]. Besides, the disadvantage of the excessive amplification of noise by equalization was overcome [25]. In some studies, the image algorithm was applied in the processing of X-ray and magnetic resonance image (MRI), and the results revealed that the image enhancement algorithm obviously improved the resolution and image quality of X-ray and MRI [26]. Sheng et al. [27] processed ultrasound images based on the wavelet transformation enhancement algorithm and applied them in the ultrasound-guided laparoscopic operation. The results pointed out that the method significantly improved the quality of ultrasound images.

As a traumatic operation, ERCP lasts for a long time and causes obvious stress reactions among patients. Hence, it is necessary to not only ensure the stability of patients' respiratory circulation but also achieve a satisfactory anesthetic effect during ERCP, which requires sedation, analgesia, no body movement, and security. The use of intraoperative neuroleptics and analgesics can significantly improve patients' discomfort and reduce the incidence of intraoperative adverse reactions and postoperative complications [28]. However, there are still some disadvantages to the sedation schemes used in clinical practice [29]. In the research, remimazolam benzenesulfonate was firstly combined with esketamine. The efficacy of the combination in ERCP was discussed, and the results demonstrated that MAP, HR, RR, and SpO_2_ of the patients in the two groups all showed an obvious descending trend from T1. MAP, HR, RR, and SpO_2_ in the observation group were reduced less significantly than those in the control group, while those in the observation group at T4 were all obviously higher than those in the control group (*P* < 0.05). The results indicated that the combination of remimazolam benzenesulfonate and esketamine could maintain the stability of hemodynamics among the patients more effectively. The results of the research showed that the comparison of operation time between the patients in the two groups had no statistical differences (*P* > 0.05). The awakening time of the patients in the control group and the observation group was 22.51 ± 2.02 minutes and 9.03 ± 1.08 minutes, respectively. The awakening time of the observation group was obviously shorter than that of the control group (*P* < 0.05). Besides, VAS scores of the patients in the control group and observation group after awakening were 3.65 ± 0.33 minutes and 1.98 ± 0.18 minutes, respectively. Obviously, the VAS score of the observation group was lower than that of the control group (*P* < 0.05). The incidence of hypotension, low oxygen saturation, and respiratory suppression in the observation group was all significantly lower than those of the control group (*P* < 0.01). The comparison of the incidence of bradycardia between the observation group and the control group showed statistical differences (*P* < 0.05). The incidence of nausea, vomiting, and chill in the control group was 6 (13.04%), 4 (8.70%), and 3 (6.52%), respectively, while those in the observation group were 3 (6.52%), 1 (2.17%), and 1 (2.17%), respectively. The incidence of nausea, vomiting, and chill in the observation group was all lower than those in the control group (*P* < 0.05). The above research results suggested that the combination of remimazolam benzenesulfonate caused the reduction in postoperative awakening time and the incidence of adverse reactions and complications, which might be caused by the effective maintenance of the stability of blood flow among ERCP patients by esketamine cycle excitability [30]. Clinical studies show that remimazolam benzenesulfonate is a water-soluble super short-acting benzodiazepine that shows no stimulating effects on vascular walls and obviously improves patients' discomforts during intravenous injection. In addition, remimazolam benzenesulfonate results in decreased body movement, sedation, and amnesia. Its anesthesia and sedation intensity is as high as that of propofol with higher security. It is pointed out in some studies that remimazolam benzenesulfonate exerts little influence on the circulation system with a small fluctuation range of blood pressure and HR and stable hemodynamics [31], which is similar to the results of the research. The combination of remimazolam benzenesulfonate and esketamine obviously reduces patients' respiratory suppression. In clinical application, propofol is characterized by a fast effect, short awakening time, and controllable anesthesia depth. However, it still has some disadvantages, such as large amounts of dosage and some adverse reactions, including obvious reduction in blood pressure, bradycardia, and apnea during deep sedation [32]. Liu et al. [33] pointed out that the sedative effect of remimazolam benzenesulfonate was obviously better than that of midazolam during the diagnosis and treatment by colonoscopy. The success rate of sedation by remimazolam benzenesulfonate, the dosage of sedatives, the inhibition of the circulation system, awakening time, and other parameters were all significantly superior to those of remimazolam benzenesulfonate. The authors pointed out that remimazolam benzenesulfonate inhibited the circulatory respiratory system more mildly with faster awakening and recovery. In the research, the combination of remimazolam benzenesulfonate and esketamine obviously reduced the incidence of adverse reactions among patients, including the intraoperative reduction in blood pressure, bradycardia, and apnea.

## 5. Conclusions

Based on the image enhancement algorithm, an effective endoscopic image processing method was established. The combination of remimazolam benzenesulfonate and esketamine in ERCP showed good security and efficacy. However, there are some disadvantages to the research. The optimized enhancement algorithm was compared with that before optimization rather than other image processing algorithms. In future studies, the established algorithm and other algorithms need to be compared and analyzed. In conclusion, the research provided a reference direction and some guiding significance for 3D endoscopic image processing and ERCP anesthesia scheme.

## Figures and Tables

**Figure 1:** Image enhancement algorithm-based endoscopic image processing procedures.

**Figure 2:** Adaptive histogram equalization depicting specific processes with limited contrast.

**Figure 3:** Comparison of PSNR values (*Y* axis) representing optimized enhanced algorithm and enhanced algorithm of 3D endoscopic images processed before and after optimization.

**Figure 4:** Comparison of DE values of 3D endoscopic images processed by the enhancement algorithms before and after optimization.

**Figure 5:** Comparison of AMBE values of 3D endoscopic images processed by the enhancement algorithms before and after optimization.

**Figure 6:** Comparison of MAP of the patients in two groups at different time points (∗ indicates that the comparison with MAP at T0 had statistical differences, *P* < 0.05; # demonstrated that the comparison with the control group showed statistical differences, *P* < 0.05).

**Figure 7:** Comparison of HR of the patients in two groups at different time points (∗ indicates that the comparison with HR at T0 had statistical differences, *P* < 0.05; # shows that the comparison with the control group had statistical differences, *P* < 0.05).

**Figure 8:** Comparison of RR of the patients in the two groups at different time points (∗ indicated the comparison with RR at T0 showed statistical differences, *P* < 0.05; # showed the comparison with the control group had statistical differences, *P* < 0.05).

**Figure 9:** Comparison of SpO_2_ of the patients in two groups at different time points (∗ indicated that the comparison with SpO_2_ at T0 showed statistical differences, *P* < 0.05; # showed that the comparison with the control group had statistical differences, *P* < 0.05).

**Figure 10:** Comparison of operation time, awakening time, and postoperative VAS score of the patients in the two groups: (a) shows the comparison of operation time and awakening time in the two groups; (b) displays the comparison of postoperative VAS scores between the two groups; ∗ indicates that the comparison with the control group has statistical differences, *P* < 0.05.

**Figure 11:** Comparison of the incidence of intraoperative adverse events of the patients in two groups (∗∗ indicates that the comparison with the control group had significant differences, *P* < 0.01; ∗ shows that the comparison with the control group shows statistical differences, *P* < 0.05).

**Figure 12:** Comparison of incidence of postoperative complications of the patients in two groups (∗ indicates that the comparison with the control group had statistical differences, *P* < 0.05).

**Table 1:** Comparison of basic information about the patients in two groups.

Names	Control group (*n* = 46)	Observation group (*n* = 46)	*P* values
Age (years old)	68.15 ± 3.96	67.62 ± 4.52	0.287
Gender (cases (%))			0.604
Male	32 (69.57)	31 (67.39)	
Female	14 (30.43)	15 (32.61)	
Percentage (kg)	60.25 ± 9.18	60.03 ± 10.22	
ASA grades (cases (%))			0.513
Grade I	19 (41.30)	21 (45.65)	
Grade II	12 (26.09)	14 (30.43)	
Grade III	15 (32.61)	11 (23.91)	
Clinical diagnosis (cases (%))			0.448
Pancreas placeholder	5 (10.87)	6 (13.04)	
Gallbladder carcinoma	4 (8.70)	3 (6.52)	
Choledocholithiasis	7 (15.22)	8 (17.39)	
Biliary stricture	25 (54.35)	23 (50.00)	
Pancreatic cancer	5 (10.87)	6 (13.04)	

## Data Availability

The data about the experiment used to support the findings of this study are available from the corresponding author upon request.
